The article "Serum Levels of PDGF, EGF, and sFlt-1 in Patients with Polycystic Ovary Syndrome and Their Predictive Effects on Pregnancy Outcomes" was retracted in 2023. Reasons: unreliable results or conclusions; concerns about the data; concerns about the peer review; concerns about the citations.

# Serum Levels of PDGF, EGF, and sFlt-1 in Patients with Polycystic Ovary Syndrome and Their Predictive Effects on Pregnancy Outcomes

**DOI:** 10.1155/2021/7118464

**Published:** 2021-10-29

**Authors:** Jiefan Gao, Yangyang Song, Donghui Wang, Dan Zhang, Xiao Huang

**Affiliations:** Department of Reproductive Medicine, Cangzhou Central Hospital, Cangzhou, Hebei 061000, China

## Abstract

Polycystic ovary syndrome (PCOS) is a neuroendocrine disease with complex etiology characterized by infrequent menstruation, follicular developmental disorders, insulin resistance, and hyperandrogenism. PCOS patients often suffer from anovulatory infertility, and even after successful pregnancy promotion, spontaneous abortion is easy to occur. At present, PCOS is mainly diagnosed by auxiliary examinations such as sex hormones and B ultrasonography, and there is a lack of specific serological markers for the diagnosis of diseases. Similarly, there is a lack of effective evaluation methods for the risk of abortion in PCOS patients. Therefore, it is extremely important to explore the factors that affect the occurrence of abortion in PCOS patients and to find specific indicators that can guide the pregnancy outcome of PCOS patients. The purpose of this study was to investigate the serum levels of platelet-derived growth factor (PDGF), epidermal growth factor (EGF), and soluble fms-like tyrosine kinase-1 (sFlt-1) in PCOS patients and analyze their predictive effects on the pregnancy outcomes of PCOS patients. The results showed that serum PDGF, EGF, and sFlt-1 levels were secreted abnormally in PCOS patients with abortion and were closely related to the pregnancy outcome of PCOS patients. The combination of the three levels has the highest value in predicting the pregnancy outcome of PCOS patients, which is worth promoting.

## 1. Introduction

Polycystic ovary syndrome (PCOS) is one of the common endocrine disorders in women of childbearing age, characterized by increased androgen and persistent anovulation. The incidence of PCOS accounts for 5%–21% of infertile women and 75%–80% of anovulatory women [1, 2]. PCOS often causes symptoms such as menstrual disorders, hirsutism, acne, obesity, acanthosis nigricans, and infertility, especially infertility has become a very difficult problem for obstetricians and gynecologists. Although there are many treatment methods, their effects are not satisfactory [3, 4]. Abortion is the main adverse pregnancy outcome in PCOS patients. A large number of studies have found that high levels of androgen in PCOS patients before pregnancy are closely related to subsequent pregnancy abortion and speculated that hyperandrogenism may be the main cause of abortion in PCOS patients [5, 6]. Platelet-derived growth factor (PDGF) is mainly produced and released by platelets, mononuclear macrophages, vascular endothelial cells, vascular smooth muscle cells, placental and embryonic cells, mesangial cells, and SV40-transformed cells. PDGF transmits information through tyrosine kinase pathway in an paracrine manner in the ovary and plays an important role in regulating oocyte growth and embryo development [7, 8]. Epidermal growth factor (EGF) is a single-chain polypeptide consisting of 53 amino acids which is mainly produced in glandular, pancreatic, thyroid, liver, oocyte, blastocyst, and other tissues. It acts in the fallopian tube and uterus through paracrine to regulate the functional activities of the ovary, such as cell proliferation and differentiation, and steroid hormone production. Besides, it may be involved in the regulation of aromatase activity in ovarian granulosa cells, which is related to the occurrence of PCOS [9, 10]. Soluble fms-like tyrosine kinase-1 (sFlt-1) is a clipped form of fms-like tyrosine kinase-1 (Flt-1) that retains the ligand-binding region but does not have tyrosine kinase activity and is an angiogenic inhibitor produced by trophoblasts during pregnancy that inhibits placental angiogenesis [11, 12]. The purpose of this study was to investigate the serum levels of PDGF, EGF, and sFlt-1 in PCOS patients and analyze their predictive effects on the pregnancy outcomes of PCOS patients. The specific report is as follows.

## 2. Materials and Methods

### 2.1. Patients

A total of 201 PCOS patients who were admitted to our hospital from March 2017 to June 2019 were selected as the research subjects, aged from 21 to 38 years old, with an average age of (28.43 ± 5.92) years old and an average BMI of (24.86 ± 6.14) kg/m^2^. The course of disease ranged from 1 to 3 years, with an average course of (2.01 ± 0.76) years. Inclusion criteria are as follows: all of them meet the PCOS criteria recommended by the Rotterdam Expert Meeting of European Society of Human Reproduction and Embryology and American Society of Reproductive Medicine in 2003: (1) Patients do not ovulate or ovulate less; (2) Hyperandrogenism, and eliminating the possibility of diseases such as androgen-secreting tumors, congenital adrenal hyperplasia, and Cushing syndrome; (3) polycystic ovary: B-ultrasonography showed that the diameter of follicles was 2∽8 mm ≥12, and/or the volume increased >10 ml; those who meet the above two criteria can be diagnosed as PCOS; patients with successful pregnancy; patients whose pregnancy outcome is spontaneous abortion or successful delivery; patients with complete clinical data. Exclusion criteria were as follows: patients with a history of adverse pregnancy outcomes; those combined with other factors that may lead to adverse pregnancy outcomes; combined with malignant tumor, cardiovascular disease, and blood system disease; untreated patients with uterine malformation, intrauterine adhesions, or hydrosalpinx; and patients with follow-up loss.

### 2.2. Research Methods

All PCOS patients were followed up for 2 years by outpatient and telephone visits from the moment when the pregnancy of PCOS patients was confirmed, and the pregnancy outcome of the patients was recorded as abortion or successful delivery. According to the pregnancy outcome, all PCOS patients were divided into an abortion group (*n* = 84) and a successful delivery group (*n* = 117).

### 2.3. Observation Indicators

When the pregnancy of the PCOS patient was confirmed, 3 ml of fasting venous blood was collected from the patient in the morning, centrifuged at 3000 r/min for 10 min to collect the serum, and stored at −20 °C until the test. Serum PDGF, EGF, and sFlt-1 levels were detected by ELISA. The relevant test kits were purchased from Shanghai ELISA Technology Co., Ltd., and were operated in strict accordance with the instructions.

Clinical baseline data such as age, parity, and body mass index (BMI) were recorded for all patients. Single factor analysis and multiple factor analysis were used to analyze the related factors affecting the pregnancy outcome of the patients. The Spearman correlation was used to analyze the correlation between serum PDGF, EGF, and sFlt-1 levels of patients and pregnancy outcomes. Then, the ROC curve was used to analyze the predictive value of serum PDGF, EGF, and sFlt-1 levels on abortion in PCOS patients.

### 2.4. Statistical Methods

The results of this experiment were statistically analyzed by SPSS 20.0 (SPSS Co., Ltd., Chicago, USA). Count data were expressed by (rate), and chi-square test was used for their comparison between groups. Measurement data were expressed by (mean ± standard deviation), and *t*-test was used for their comparison between groups. Multivariate analysis adopts multiple logistic regression model. Spearman correlation analysis was used for correlation analysis. The ROC curve was used to analyze the predictive value of serum PDGF, EGF, and sFlt-1 levels for abortion in PCOS patients. *P* < 0.05 indicates that the difference is statistically significant.

## 3. Results

### 3.1. Comparison of Serum PDGF, EGF, and sFlt-1 Levels between the Two Groups

The levels of serum PDGF and EGF in the abortion group were higher than those in the successful delivery group, and the level of sFlt-1 was lower than that in the successful delivery group (*P* < 0.05), as shown in Figure 1.

### 3.2. Analysis of Single Factor Affecting Pregnancy Outcome of PCOS Patients

Univariate analysis showed that age, BMI, diabetes, hypertension, endometrial thickness, and serum PDGF, EGF, and sFlt-1 levels were all related to the pregnancy outcome of PCOS patients (*P* < 0.05), as shown in Table 1.

### 3.3. Analysis of Multiple Factors Affecting Pregnancy Outcome of PCOS Patients

Multivariate logistic analysis showed that age, BMI, diabetes, hypertension, endometrial thickness, and serum PDGF, EGF, and sFlt-1 levels were all independent factors affecting the pregnancy outcome of PCOS patients (*P* < 0.05), as shown in Tables 2 and 3.

### 3.4. Analysis of Correlation between Serum PDGF, EGF, sFlt-1 Levels and Pregnancy Outcomes of PCOS Patients

Spearman correlation analysis showed that serum PDGF and EGF levels were positively correlated with the pregnancy outcome of PCOS patients (*r* = 0.694, *r* = 0.725, *P* < 0.001), and serum sFlt-1 level was negatively correlated with the pregnancy outcome of PCOS patients (*r* = −0.586, *P* < 0.001), as shown in Table 4.

### 3.5. Prediction Value of Serum PDGF, EGF, and sFlt-1 Levels in the Pregnancy Outcome of PCOS Patients

The AUC of serum PDGF for predicting pregnancy outcome in PCOS patients was 0.757 (95% CI: 0.657–0.857), and when the optimal cutoff value was 2811.61 ng/L and the Youden index was 0.488, the sensitivity and specificity were 69.7% and 79.1%, respectively. The AUC of serum EGF level for predicting the pregnancy outcome of PCOS patients was 0.795 (95% CI: 0.705–0.884). When the optimal cutoff value was 115.71 ng/L and the Youden index was 0.428, the sensitivity and specificity were 72.7% and 70.1%, respectively. The AUC of serum sFlt-1 for predicting the pregnancy outcome of PCOS patients was 0.737 (95% CI: 0.634–0.840), and when the optimal cutoff value was 68.91 ng/L and the Youden index was 0.382, the sensitivity and specificity were 60.6% and 77.6%, respectively. The AUC for the combined prediction of pregnancy outcome in PCOS patients was 0.876 (95% CI: 0.802–0.950). When the Youden index was 0.654, the sensitivity and specificity were 81.8% and 83.6%, respectively, as shown in Table 5 and Figure 2.

## 4. Discussion

PCOS is a neuroendocrine disease with complex etiology characterized by infrequent menstruation, follicular developmental disorders, insulin resistance, and hyperandrogenism. PCOS patients often suffer from anovulatory infertility, and even after successful pregnancy promotion, spontaneous abortion is easy to occur [13–16]. At present, PCOS is mainly diagnosed by auxiliary examinations such as sex hormones and B ultrasonography, and there is a lack of specific serological markers for the diagnosis of diseases. Similarly, there is a lack of effective evaluation methods for the risk of abortion in PCOS patients [17, 18]. Therefore, it is extremely important to explore the factors that affect the occurrence of abortion in PCOS patients and to find specific indicators that can guide the pregnancy outcome of PCOS patients. PDGF is a major mitogen and chemokine in the body, and it is a homologous or heterologous dimer consisting of four peptide chains (A, B, C, and D chains). It was mainly divided into four regions: signal region, extracellular region, transmembrane region, and intracellular region. The intracellular part contained tyrosine kinase and tyrosine phosphate. PDGF receptor is a membrane glycoprotein that is distributed in many cells, such as ovarian foam cells and granulosa cells, fibroblasts, glial cells, smooth muscle cells, lipid storage cells, osteoblasts, endothelial cells, and so on. PDGF is present in granulosa cells of follicles, as well as in ova and antral follicles [19, 20]. PDGF stimulates the growth of vesicle membrane cells and inhibits the secretion of progesterone and androstenedione stimulated by luteinizing hormone (LH). It plays an important role in follicular development and growth in the body. PDGF cannot exert its biological effects until it binds to the corresponding receptor on the cell membrane. High-degree close binding of PDGFA and B chains to PDGFR has been observed in pig eggs and granulosa cells. PDGF is chemically stable and resistant to high temperature. Previous studies have shown that PDGF can regulate the growth of follicles, and its receptor exists in both granulosa cells and ova. As mentioned above, PDGF works by binding to receptors in the ovary to modify the FSH-cAMP pathway of ovarian granulosa cells, resulting in enhanced aromatase activity and thus increased estrogen secreted by the granulosa cells [21, 22].

EGF receptor (EGFR) has protein kinase activity specific for tyrosine residues, which phosphorylates intracellular tyrosine residues and interacts with two intracellular messenger pathways (cAMP messenger pathway and phosphoinositide metabolic messenger pathway) to produce biological effects. In human ovary, EGF was highly expressed in primordia and preantral follicles, and in granulosa cells of preantral follicles, follicular membranes of all levels of follicles, atretic follicles, and luteal cell membrane. There is evidence that EGF is mainly produced by foam membrane cells and plays a paracrine regulatory role in nearby granulosa cells. It regulates the activity of granulosa cells by stimulating the production of progesterone expressed by follicle-stimulating hormone (FSH) receptor and inhibits the synthesis of *E*_2_ and inhibin to promote the production of progesterone [23, 24]. sFlt-1 is a modified soluble receptor that can bind to vascular endothelial growth factor A (VEGF-A), reduce VEGF production, hinder the binding of VEGF to membrane receptor Flt-1 and antagonize VEGF-mediated endothelial protection, and inhibit its angiogenic effect, causing endothelial damage. It can also be used on follicles and affect the growth of follicles, which in turn affect the normal function of the ovary [25, 26].

The results of this study showed that serum PDGF and EGF levels in the abortion group were higher than those in the successful delivery group, and sFlt-1 level was lower than that in the successful delivery group. These results indicated that serum levels of PDGF, EGF, and sFlt-1 were abnormally secreted in aborted PCOS patients. In addition, Spearman's correlation analysis showed that serum PDGF and EGF levels had a positive correlation with the pregnancy outcome of PCOS patients, and serum sFlt-1 levels had a negative correlation with the pregnancy outcome of PCOS patients. These results indicated that serum levels of PDGF, EGF, and sFlt-1 were closely related to the pregnancy outcome of PCOS patients. The analysis showed that under normal conditions, the local cytokines of ovary maintained dynamic balance, and a small amount of PDGF existed in human body. When the local androgen of ovary increased to a certain threshold, the secretion of PDGF was increased, the activity of aromatase was enhanced by modifying FSH-cAMP pathway, and the conversion of androgen to estrogen was promoted. The increased concentration of estrogen promotes the increased secretion of EGF, which inhibits the activity of aromatase through the FSH-cAMP pathway and reduces the conversion of androgen. On the one hand, sFlt-1 can negatively regulate VEGF and block oocyte maturation; on the other hand, it acts on steroid hormones to affect androgens in the granular cell layer, indirectly interfering with estrogen expression and disrupting ovarian function, thus promoting the occurrence of PCOS [27, 28].

The results of univariate and multivariate analyses in this study showed that age, BMI, diabetes, hypertension, endometrial thickness, and serum PDGF, EGF, and sFlt-1 levels were all independent factors affecting the pregnancy outcome of PCOS patients. The causes were analyzed as abnormal fetus genes and increased abortion probability due to special physiological reasons of elderly parturients, such as reproductive system function degradation, poor body quality, endocrine deficiency, and overwork. Therefore, nutrition supplement during pregnancy should be strengthened to improve the body quality of elderly PCOS patients so as to reduce the probability of abortion. Obesity during pregnancy will cause placental and structural and functional abnormalities or even inflammatory reactions, which is not conducive to the development of the embryo, so its abortion rate is high. Therefore, during the treatment and pregnancy, a scientific and reasonable diet menu and reasonable exercise should be made for them, so as to control their weight in an appropriate range and reduce the rate of abortion. Hyperglycemia and hypertension are complications of pregnancy. Hypertension can cause abnormal or undeveloped fetus. Hyperglycemia can cause hydramnios and macrosomia, which are not conducive to fetal development. Therefore, blood pressure and blood sugar should be controlled before pregnancy to avoid affecting the outcome of pregnancy. Endometrium is the implantation site and the supply station of embryo nutrition. With a thin endometrium, the embryo implantation is not only difficult, but also the probability of abortion is high. Therefore, pregnancy preparation should be targeted treatment, in order to reduce its abortion rate.

The results of ROC curve in this study showed that the AUC of serum PDGF, EGF, and sFlt-1 to predict the pregnancy outcome of PCOS patients was 0.757, 0.795, and 0.737, respectively, and the AUC of the three combined to predict the pregnancy outcome of PCOS patients was 0.876. These results indicated that the combined use of serum PDGF, EGF, and sFlt-1 levels in the prediction of pregnancy outcomes in PCOS patients was significantly superior to the single prediction and had higher prediction value. Therefore, the combined detection of serum PDGF, EGF, and sFlt-1 levels in PCOS patients can timely evaluate the condition and give treatment, which is conducive to improving the pregnancy situation and the successful delivery rate of patients.

## 5. Conclusion

Serum PDGF, EGF, and sFlt-1 levels are abnormally secreted in aborted PCOS patients and are closely related to the pregnancy outcome of PCOS patients. The combination of the three factors has the highest value in predicting the pregnancy outcome of PCOS patients and is worthy of promotion. Age, BMI, diabetes, hypertension, endometrial thickness, and serum PDGF, EGF, and sFlt-1 levels were all independent factors influencing the pregnancy outcome of PCOS patients.

## Figures and Tables

**Figure 1:** Comparison of serum PDGF, EGF, and sFlt-1 levels between the two groups. ^*∗*^*P* < 0.05.

**Figure 2:** ROC curve of serum PDGF, EGF, and sFlt-1 levels predicting pregnancy outcome of PCOS patients.

**Table 1:** Analysis of single factor affecting pregnancy outcome of PCOS patients.

Factor	*n*	Successful delivery group (*n* = 117)	Abortion group (*n* = 84)	*t/χ* ^2^	*P*
Age (year)	201	29.63 ± 5.82	27.57 ± 6.05	2.419	0.017
Parity				1.289	0.256
Primiparity	165	93 (79.49)	72 (85.71)		
> 1 time	36	24 (20.51)	12 (14.29)		
BMI (kg/m^2^)				5.419	0.019
< 25	153	96 (82.05)	57 (67.86)		
≥ 25	48	21 (17.95)	27 (32.14)		
Diabetes				5.029	0.025
Yes	18	6 (5.13)	12 (14.29)		
No	183	111 (94.87)	72 (85.71)		
Hypertension				4.806	0.028
Yes	30	12 (10.26)	18 (21.43)		
No	171	105 (89.74)	66 (78.57)		
Endometrial thickness (mm)				5.027	0.025
≥ 5 mm	68	47 (40.17)	21 (25.00)		
< 5 mm	133	70 (59.83)	63 (75.00)		
Treatment				0.133	0.715
Operation	76	43 (36.75)	33 (39.29)		
Medicines	125	74 (63.25)	51 (60.71)		
PDGF (ng/L)	201	3182.31 ± 217.65	3290.66 ± 251.94	3.258	0.001
EGF (ng/L)	201	108.40 ± 8.67	112.20 ± 10.34	2.826	0.005
sFlt-1(ng/L)	201	64.69 ± 15.29	56.85 ± 16.05	3.512	0.001

**Table 2:** Assignment for multivariate analysis of factors.

Factors	Variable	Assignment
Age	X1	Continuous variable
BMI	X2	< 25 = 0, ≥25 = 1
Diabetes	X3	No = 0, Yes = 1
Hypertension	X4	No = 0, Yes = 1
Endometrial thickness	X5	≥ 5 = 0, <5 = 1
PDGF	X6	Continuous variable
EGF	X7	Continuous variable
sFlt-1	X8	Continuous variable

**Table 3:** Analysis of multiple factors affecting pregnancy outcome of PCOS patients.

Variables	*B*	SE	Wald *γ*^2^	*P*	OR	95% CI
Age	1.284	0.357	12.649	<0.001	3.611	1.805–7.296
BMI	0.876	0.394	5.315	0.021	2.401	1.085–4.693
Diabetes	1.815	0.731	6.291	0.012	6.141	1.592–22.741
Hypertension	0.788	0.297	5.435	0.019	2.199	1.206–3.982
Endometrial thickness	1.419	0.425	11.273	< 0.001	4.133	1.915–12.624
PDGF	0.806	0.305	6.802	0.009	2.239	1.238–4.054
EGF	0.917	0.408	5.072	0.024	2.502	1.127–5.554
sFlt-1	-0.589	0.251	5.562	0.018	0.555	0.340–0.905

**Table 4:** Analysis of correlation between serum PDGF, EGF, sFlt-1 levels and pregnancy outcomes of PCOS patients.

Predictive indexes	Pregnancy outcomes	
	*r*	*P*
PDGF	0.694	< 0.001
EGF	0.725	< 0.001
sFlt-1	−0.586	< 0.001

**Table 5:** Prediction value of serum PDGF, EGF, and sFlt-1 levels in the pregnancy outcome of PCOS patients.

Predictive indexes	AUC	95%CI	Youden index	Sensitivity (%)	Specificity (%)	Cutoff value
PDGF	0.757	0.657–0.857	0.488	69.7	79.1	2811.61 ng/L
EGF	0.795	0.705–0.884	0.428	72.7	70.1	115.71 ng/L
sFlt-1	0.737	0.634–0.840	0.382	60.6	77.6	68.91 ng/L
Combined predictive	0.876	0.802–0.950	0.654	81.8	83.6	—

## Data Availability

The data used to support the findings of this study can be obtained from the corresponding author upon reasonable request.
